# A Multiperson Pose Estimation Method Using Depthwise Separable Convolutions and Feature Pyramid Network

This article has been retracted.

**DOI:** 10.1155/2021/6903895

**Published:** 2021-12-15

**Authors:** Qidong Du

**Affiliations:** Educational Technology Center, Guangzhou Railway Polytechnic, Guangzhou, Guangdong 510430, China

## Abstract

In the process of multiperson pose estimation, there are problems such as slow detection speed, low detection accuracy of key point targets, and inaccurate positioning of the boundaries of people with serious occlusion. A multiperson pose estimation method using depthwise separable convolutions and feature pyramid network is proposed. Firstly, the YOLOv3 target detection algorithm model based on the depthwise separable convolution is used to improve the running speed of the human body detector. Then, based on the improved feature pyramid network, a multiscale supervision module and a multiscale regression module are added to assist training and to solve the difficult key point detection problem of the human body. Finally, the improved soft-argmax method is used to further eliminate redundant attitudes and improve the accuracy of attitude boundary positioning. Experimental results show that the proposed model has a score of 73.4% in AP on the 2017 COCO test-dev dataset, and it scored 86.24% on PCKh@0.5 on the MPII dataset.

## 1. Introduction

Human body pose estimation is based on human bone joint points (key points) as the research object by detecting the position information of the joint points, estimating the connection between the joint points, and then reconstructing the method of human limbs [1]. It is the basic link to realize tasks such as behavior recognition [2, 3], posture tracking [4, 5], image generation [6], human-computer interaction [7], and emotion recognition [8], and related research has received extensive attention. However, due to crowded background, body occlusion, motion blur, invisible key points, etc., human pose estimation is very challenging. Early human pose estimation relied on hand-labeled features. The pose estimation is expressed as a tree structure or graphical model, which fails to effectively deal with the spatial structure relationship between key points. The robustness of attitude estimation detection is poor. With the development of the convolutional neural network (CNN) in the field of human pose estimation, the performance of key point detection has been greatly improved.

Multiperson posture estimation based on deep learning has gone through the development process of direct regression coordinates to predicting heat maps. Regarding the direct return to the coordinate method, as early as 2014, Toshev and Szegedy [9] proposed DeepPose. It introduces CNN with powerful fitting ability into the field of pose estimation and forcibly returns the coordinates of key points of human pose. By 2015, Fan et al. [10] proposed a dual-source CNN, which introduced local representation and overall vision, and added prior knowledge to the network. However, the use of direct coordinate regression is prone to overfitting. On this issue, stacked hourglass network (SHN) [11] and feature pyramid network (FPN) [12] have emerged as representative heat map solutions, which have obvious advantages. The FPN method can obtain different semantic information. However, due to the lack of the contextual information intercommunication mechanism, as the area Intersection of Union (IoU) increases, the detection performance decreases. Applied to human body posture, it is not conducive to key point detection. Baseline [13] used the improved residual block to predict the heat map of key points with multiscale features but did not eliminate redundant postures. Fang et al. [14] proposed the regional multiperson pose estimation (RMPE) model. The spatial transformation network (STN) is used to extract the human body region frame to improve the overall performance of the model. However, in the RMPE model, when the key points of the human body are occluded, the detection rate needs to be improved. In addition, the number of inspectors has a greater impact on the inspection time, and the model runs slowly.

For this reason, this paper proposes a multiperson pose estimation method based on depthwise separable convolution and feature pyramid network. This method uses YOLOv3 as the human target detection model and combines it with the depthwise separable convolution which can reduce the parameter scale. It effectively improves the target detection speed. By improving the feature pyramid network and adding a multiscale supervision module and a multiscale regression module to assist training, a Gaussian heat map is generated. It also searches and locates key points to improve the robustness of positioning difficult key points. Finally, the improved soft-argmax method is used to find the best pose target bounding box and eliminate redundant poses. Experiments show that the method in this paper has a small amount of parameters and has strong detection performance.

## 2. Materials and Methods

### 2.1. Network Architecture

The method proposed in this paper belongs to the top-down framework. The overall method network structure is shown in Figure 1.

The first part is human target detection. The model is improved after replacing the standard convolution structure of the original YOLOv3 model network with the depthwise separable convolution structure. The second part is to improve the feature pyramid network. Multiscale supervision module and multiscale regression module are added to assist training to detect and classify key points. The third part is the use of improved soft-argmax technology to extract the coordinates of key points in the heat map.

### 2.2. Depthwise Separable Convolution YOLOv3 Model

The YOLOv3 detection method is one of the excellent algorithms in the field of target detection. The feature acquisition is achieved through the standard convolution structure of the convolution kernel. The standard convolution structure (Figure 2(a)) is to perform convolution operations on each channel of the input data with a specific convolution kernel, and it is the process of adding up the convolution results of each channel. When the number of channels is too large, the number of convolution kernels will become huge, resulting in a decrease in the calculation rate. The depthwise separable convolution (DSC) [15] is the product of splitting the standard convolution structure. In its structure (Figure 2(b)), the convolution operation is decomposed into a separate convolution process and a point convolution process. That is, each channel of the input data performs a deep convolution operation and then uses a point convolution to linearly connect the output of the deep convolution. This network structure can greatly reduce the model parameters. Therefore, the detection rate can be increased when the detection accuracy has not changed.

There is an image of *W* × *H* × *C* with a channel number of *C* and a convolution kernel 3 × 3. The padding pixel is set to 1, and the stride is set to 1. The feature map of each channel is obtained by a separate convolution operation. The parameters of standard convolution and depthwise separable convolution are shown in equations (1) and (2), respectively:

(1) $$\begin{array}{c} P_{1}=3\times 3\times C\times K, \end{array}$$

(2) $$\begin{array}{c} P_{2}=3\times 3\times C+1\times 1\times K. \end{array}$$

The multiplication operations of the standard convolution and depthwise separable convolution are shown in equations (3) and (4), respectively:

(3) $$\begin{array}{c} C_{1}=H\times W\times C\times K\times 3\times 3, \end{array}$$

(4) $$\begin{array}{c} C2=H\times W\times C\times 3\times 3+H\times W\times C\times K. \end{array}$$

It can be seen from *P*_1_ > *P*_2_ and *C*_1_ > *C*_2_ that the depthwise separable convolution is smaller than the standard convolution in terms of the amount of parameters and the amount of multiplication operations.

### 2.3. Improved Feature Pyramid

In order to improve the low-level semantic features such as texture and shape of the detected key points and enhance the search performance of the key points that are difficult to detect the pose, an improved feature pyramid network model is used [16]. The model will be able to generate multiple feature channels of the same scale output mapping and locate them in the same network stage, which is defined as a pyramid network layer. Its network structure is shown in Figure 3.

#### 2.3.1. Parallel Residual Layer

Parallel residual layer (PRL) is an important detector to improve the feature pyramid. Based on the standard feature pyramid, 3 × 3 convolution is added in the horizontal direction. The branch structure of the multiscale convolution [17] is used to eliminate the influence of aliasing and obtain uniform features. The difficult samples are detected by expanding the receptive field. The number of compressed channels is used to obtain the characteristics of high resolution and strong semantic information. Finally, combined with the context, the key point information that is difficult to detect is judged.

As shown in Figure 3, the output characteristics of conv2, conv3, conv4, and conv5 are denoted as *C*_1_, *C*_2_, *C*_3_, and *C*_4_, respectively. The first step is to extract the features of the input image and establish four convolution features with different resolutions and channel numbers. In the second step, in the order from top to bottom, the {*C*_4_, *C*_3_, *C*_2_, *C*_1_} four-layer network characteristics are taken, more than 2 times the sampling is performed, and the number of channels is compressed to 256 dimensions. The third step is to take the characteristics of the {*C*_3_, *C*_2_, *C*_1_} three-layer network and perform 1 × 1 convolutional dimensionality reduction processing. The compressed channel is also 256 dimensions. In the fourth step, after repeating the second and third steps, the features of the sampling model are used to calculate the three-layer features. In the fifth step, the new feature pyramid is obtained by improving the feature pyramid formula [16] of the top features of the fourth and second steps. Suppose the input feature is *x* and the corresponding network weight is *W*, the convolution function is ℱ(*·*), the upsampling is *U*(*·*), the activation function is *σ*(*·*), the number of branches is *N*, and the convolution kernel bias is *b*. The output characteristics of the parallel residual layer are shown in the following formula:

(5) $$\begin{array}{c} y={ℱ}_{\text{PRL}}\left(x\right)=U\left(\sigma \sum_{i=1}^{N}W_{i}x_{i}+x+b\right). \end{array}$$

The framework of the parallel residual network layer in this paper is shown in Figure 4. Its structure is mainly composed of two residual blocks. [*d*, *w*_*c*_, *h*_*c*_] is the input feature of the *c*th layer. The parallel residual layer can ensure that the output feature maps of different convolution operations have the same size, so as to facilitate feature splicing.

The first residual block is composed of the bottleneck module [18]. Its structure includes three convolutional layers, a normalization layer, and an activation layer. Among them, the first 1 × 1 convolution kernel is used for feature dimension reduction, reducing the number of channels. The second 3 × 3 convolution kernel is used for feature downsampling, effectively training data and extracting features. The third 1 × 1 convolution kernel is used to increase the dimension of the feature and restore the original dimension of the feature. The second residual module is composed of 3 convolutional layers, normalization layer, activation layer, and upsampling layer. The branch output results of the two residual blocks are connected to the residuals to obtain new features. Finally, feature stitching is performed.

#### 2.3.2. Multiscale Supervision and Multiscale Regression

By combining the features obtained from the context information of the feature pyramid, the function of the heat map of the classification key points is realized. In order to further improve the utilization of global information, a multiscale supervision model (MSS model) [19] is added to achieve the purpose of deconvolution for supervision. In order to calculate the residual difference between the real heat map and the predicted heat map, a 1 × 1 convolution is used. The high-dimensional features are reduced in dimensionality, and the mapping is transformed into features with the required number of channels. The number of channels in the heat map is the same as that of key points on the human body. At the same time, the downsampling method is adopted so that the real key point heat map of the human body can match the key point prediction heat map at each scale. The specific structure is shown in Figure 3.

In order to optimize the result, the loss function *L*_MSE_ is set. *L*_MSE_ is the mean value of the mean square error (MSE) between the predicted heat map and the real heat map. Among them, the real heat map generates a two-dimensional Gaussian distribution centered on the real coordinates of each key point, denoted as *G*_*k*_^*d*^(*x*, *y*), as shown in the following formula:

(6) $$\begin{array}{c} G_{k}^{d}\left(x,y\right)=\frac{1}{2\pi \theta^{2}}\exp\left\{\frac{-\left[{\left(x-x_{k}\right)}^{2}+{\left(y-y_{k}\right)}^{2}\right]}{2\sigma^{2}}\right\}. \end{array}$$

Among them, *d* (*d* = 1, 2, and 3) represents the number of scales. *k* represents the first few key points. (*x*, *y*) stands for pixel coordinates. (*x*_*k*_, *y*_*k*_) represents the real coordinates of the *k*th key point. *σ* represents the standard deviation of the Gaussian distribution, and it controls the radial range of the function. *K* represents the total number of key points of the body. The predicted heat map is denoted as *P*_*k*_^*d*^(*x*, *y*). The loss function *L*_MSE_ can be defined as

(7) $$\begin{array}{c} L_{\text{MSE}}=\frac{1}{3K}\overset{3}{\underset{d=1}{\sum }}d\cdot \left[\overset{K}{\underset{k=1}{\sum }}\underset{x,y}{\sum }{\left\|P_{k}^{d}\left(x,y\right)-G_{k}^{d}\left(x,y\right)\right\|}_{2}^{2}\right]+\frac{3}{K}\overset{K}{\underset{k=1}{\sum }}\underset{x,y}{\sum }{\left\|P_{k}^{4}\left(x,y\right)-G_{k}^{3}\left(x,y\right)\right\|}_{2}^{2}. \end{array}$$

In order to improve the consistency of the estimated pose structure, a multiscale regression module (MSR module) is used to globally optimize the key point heat map. The multiscale heat map after feature stitching is used as the input. After 1 × 1 convolution, the heat maps on all scales are fused to refine the estimated posture.

### 2.4. Soft-Argmax Regression

After the above network reasoning, in order to ensure end-to-end differentiability, soft-argmax [20, 21] is used to replace the traditional nonmaximum suppression (NMS) to select the extreme point position and obtain the key point heat map coordinates. The heat map of the key points is normalized, and the weighted sum is in the interval [0, 1]. From equation (8), we can see that *M* × *H* is the size of the heat map. If *G*_*k*_(*x*, *y*) is 0 or 1, there are a lot of values close to 0 in the heat map. The availability of the 0 value will affect the accuracy of the regression to a certain extent.

(8) $$\begin{array}{c} S_{k}\left(x,y\right)=\frac{e^{G_{k}\left(x,y\right)}}{\sum_{x}^{M}\sum_{y}^{H}e^{G_{k}\left(x,y\right)}}. \end{array}$$

To this end, the introduction of *λ* coefficient is to adjust *G*_*k*_(*x*, *y*), as shown in the following formula:

(9) $$\begin{array}{c} S_{k}\left(x,y\right)=\frac{e^{\lambda G_{k}\left(x,y\right)}}{\sum_{x}^{M}\sum_{y}^{H}e^{\lambda G_{k}\left(x,y\right)}}. \end{array}$$

In general, the default value of *λ* is 1, which does not affect the original soft-argmax regression. For the soft-argmax regression effect is not obvious, *λ* is manually set to improve the final prediction accuracy of the pose.

## 3. Experiment and Analysis

Experimental environment: the operating system is Ubuntu16.04, 64-bit operating system, the CPU environment is i7-4770k, the memory is 32 G, and 512 G SSD + 1T 7200 SATA 3.5. The GPU environment is NVIDIA Quadro P2000 5 GB. The training environment is PyTorch + Python 3.6.

### 3.1. Dataset and Evaluation Indicators

Two public benchmark datasets, COCO dataset and MPII dataset, are used to train and test the proposed method. The MPII dataset includes annotated pictures of more than 40,000 people. The human body sample is represented by 16 key points. The COCO dataset has 57,000 images containing 15,000 human instances. The number of key points is 17.

Inputting the image scale in the network, the corresponding COCO dataset is 256 × 192 and 384 × 288, and MPII is 256 × 256. The mean value of the image preprocessing parameters *M* = [0.485, 0.456, 0.406], and the standard deviation *S* = [0.229, 0.224, 0.225]. With the human body as the center, random rotation (−45°, +45°), zoom (−30%, +30%), and flipping are used.

COCO dataset evaluation indicators: average precision (AP) and average recall (AR) based on object keypoint similarity (OKS) are used as the main evaluation indicators of the experiment.

Evaluation index of the MPII dataset: head normalized percentage of correct keypoints (PCKh) is used as the experimental evaluation index.

### 3.2. Experimental Results and Analysis

A comparative experiment on the COCO dataset is carried out. DeepPose [9], SHN [11], FPN [12], baseline [13], and the method in this article are used to test each joint on the COCO test set. The output results are visually compared, as shown in Figure 5.

It can be seen that DeepPose [9] using coordinate regression failed to estimate the complete posture. SHN [11] and FPN [12] failed to accurately detect the shoulders, wrists, etc., occluded by the image. Attitude redundancy appeared during baseline [13] detection. The improved network has a better detection effect on “difficult points” in a complex environment and is better than other methods on the whole.

In order to evaluate the performance of the multiperson pose estimation method, the method in this paper is compared with DeepPose, SHN, FPN, baseline, and other algorithms on the COCO dataset.

It can be seen from Table 1 that DeepPose relies on coordinate regression, and the learned filter captures the pose attributes at a rough scale. The network's ability to view details is limited and is not sufficient to accurately locate body joints at all times. Compared with DeepPose, the method in this paper improves AP and AR by 6.9% and 5.3%, respectively. Compared with the SHN method and FPN method, the algorithm in this paper improves AP and AR by 5.1%, 8.8%, 5.1%, and 3.2%, respectively. Baseline introduces a multiscale supervision module and a multiscale regression module. The novel coordinate extraction method also effectively improves the performance of the model. However, it ignores the fusion between high-level features and bottom-level features. As a result, all dimensional feature maps cannot be fully utilized, and the detection accuracy rate is not a better value. This algorithm directly uses the heat map, which reduces the error caused by coordinate regression conversion. In this paper, AP and AR reached 73.4% and 78.6%, respectively.

Under the same experimental environment, the efficiency of SHN and FPN algorithms is compared. As shown in Table 2, when the number of iterations is the same, average processing time, giga floating-point operations, and the number of parameters on the COCO test set are compared. Compared with the SHN model algorithm, the average processing time of this method is 25 ms. The model parameters account for about 1/3 of it, which meets the requirements of real-time detection. In addition, although the FPN model algorithm has higher detection accuracy, it also has the problem of increased complexity.

In the COCO dataset, some scenes are selected, and the scenes have different degrees of occlusion with everyone. The method in this paper can accurately estimate the position of each joint. It is verified that the method in this paper has a good positioning effect for multiperson pose boundary estimation, as shown in Figure 6.

### 3.3. Ablation Experiment

On the MPII dataset, the PCKh evaluation criteria are set, including the head, shoulder, elbow, wrist, hip, knee, and ankle. Its threshold *r* is set to 0.5. The impact of different modules on the performance of the method is analyzed, and the results are shown in Table 3. Compared with the FPN model, the increase of PRL in the network increases the PCKh@0.5 index by 0.67%. The elbow, wrist, hip, knee, and ankle increased by 0.56%, 1.54%, 0.42%, 0.42%, and 0.26%, respectively. On this basis, MSS and MSR are added to the network, and the detection indicators in difficult-to-detect parts are significantly improved. For example, the elbow, wrist, knee, and ankle have increased by 1.51%, 1.75%, 1.18%, and 1.82%, respectively. With the addition of soft-argmax on the basis of MSS and MSR, the elbow, wrist, knee, and ankle increased by 0.05%, 0.12%, 0.80%, and 0.40%, respectively. It shows that the use of soft-argmax to select the extreme point position and obtain the key point coordinates of the heat map has a certain effect in solving the problem of lack of accuracy.

## 4. Conclusions and Future Works

This paper follows a top-down scheme and proposes a multiperson pose estimation method using depthwise separable convolution and feature pyramid network. Using the depthwise separable convolution YOLOv3 model as a human body detector is beneficial to improve the speed of multiperson pose detection. Based on the parallel residual network, it is helpful to expand the receptive field to detect difficult samples and obtain high resolution and strong semantic information features. The fusion of high-level and low-level features through multiscale supervision and multiscale regression is conducive to solving the difficult key point detection problem of the human body. The improved soft-argmax method is used to improve the accuracy of attitude boundary positioning. The experimental results on the 2017 COCO test-dev and MPII datasets show that this paper has certain advantages in accuracy compared with recent multiperson pose estimation algorithms. In human body pose estimation, higher accuracy often requires more complex networks as support. Using new methods to reduce complexity, optimize network reasoning speed, strengthen network generalization ability, and adaptively control network parameters is the next step of this paper.

## Figures and Tables

**Figure 1:** Schematic diagram of the overall method network structure.

**Figure 2:** Comparison of the (a) standard convolution and (b) depthwise separable convolution.

**Figure 3:** Improved feature pyramid network structure.

**Figure 4:** Network framework of parallel residual layers.

**Figure 5:** Comparative experimental results of different algorithms in COCO datasets. (a) DeepPose [9]. (b) SHN [11]. (c) FPN [12]. (d) Baseline [13]. (e) This work.

**Figure 6:** Qualitative results of some example images in COCO datasets.

**Table 1:** Comparison of different methods' results in COCO datasets.

Methods	AP	AP^@50^	AP^@75^	AP^@M^	AP^@L^	AR
DeepPose	66.5	79.6	72.6	62.4	71.7	73.9
SHN	68.3	84.4	68.8	65.4	77.5	69.8
FPN	68.3	84.4	78.8	65.4	77.5	75.4
Baseline	71.8	87.5	79.3	68.1	78.3	77.2
This work	73.4	87.8	79.2	68.4	77.5	78.6

**Table 2:** Comparison of model efficiency.

Methods	Average processing time (ms)	GFLOPs/(10^9^ times)	Number of parameters
SHN	64	20.2	4.7 × 10^7^
FPN	22	6.4	1.4 × 10^7^
This work	25	6.9	1.5 × 10^7^

**Table 3:** Comparison of results of different components on the MPII dataset.

Methods	Head	Shoulder	Elbow	Wrist	Hip	Knee	Ankle	Mean
FPN	94.42	93.48	84.81	79.53	84.11	78.92	73.87	84.16
+PRL	94.87	94.52	85.37	81.07	84.53	79.34	74.13	84.83
+MSS and MSR	94.89	95.31	86.88	82.82	85.93	80.52	75.95	86.04
+Soft-argmax	94.89	95.31	86.93	82.94	85.96	81.32	86.35	86.24

## Data Availability

The data included in this paper are available without any restriction.
